# Continuous Use Intention of Mobile Social Network Information Service Based on User Behavior Perception

**DOI:** 10.1155/2022/3050180

**Published:** 2022-04-16

**Authors:** Jingjing Lv, Nan Wang, Yin Ye, Wenhe Li

**Affiliations:** ^1^School of Economics, Guangdong Ocean University, Zhanjiang 524088, China; ^2^School of Management, Guangdong Ocean University, Zhanjiang 524088, China

## Abstract

In order to improve the willingness of continuous use of mobile social network information services, this study combines user behavior perception to analyze the continuous use of mobile social network information services and proposes a data coverage optimization strategy based on service quality perception. Furthermore, this study measures participants' regional preferences based on the duration of participants in the perceptual region and the number of historical perceptual tasks completed on the perceptual region. In addition, this study designs a perceptual data coverage optimization algorithm to optimize the perceptual data coverage and ensure the real-time validity of the perceptual data. Through algorithm research and systematic evaluation, it can be seen that the continuous use willingness system of mobile social network information service based on user behavior perception can basically meet the actual needs.

## 1. Introduction

There are many classification methods for mobile location services, including the method of dividing according to whether the positioning is required, the method of dividing according to the service request method, the method of dividing according to the current location positioning, etc. However, by far, the most common method is the classification of mobile location services according to service usage. According to the service usage, mobile location services can be divided into two categories: personal applications and industry applications. Mobile transaction service is based on positioning technology, and users conduct e-commerce transactions through mobile payment. The main mode of mobile location service in the field of industrial applications is to determine the specific location of the user through positioning technology, so as to realize monitoring or scheduling and other work applications. It mainly includes emergency rescue service, vehicle monitoring and dispatching, personnel dispatching, and other functions.

LBSNS (location-based social networking service) is a service function project that integrates the two functions of “location” and “social networking.” It can be translated as “mobile location social network service” or “social network location service.” At present, there is no unified translation noun in academic research. The difference between LBSNS and browsing social networking sites anytime and anywhere through mobile clients such as mobile phones is that it highlights the win-win meaning of location and social networking. By determining their location in the software, users can actively publish and share them on social platforms. They can not only find nearby friends by location but also search for discount information of nearby businesses and inquire about the latest activities and services of various businesses that cooperate with social networking sites.

This study analyzes the willingness to use mobile social network information services based on user behavior perception and combines the intelligent model to provide a theoretical reference for the follow-up research on the willingness to use mobile social network information services.

## 2. Related Work

In the research field of LBS application mode, scholars have discussed LBSNS from different perspectives: Du Liting analyzed the mode and function of mobile social network services, as well as the communication characteristics from the perspective of communication, to provide research on the development of the commercial value of LBSNS. It has a certain reference significance [1]. Literature [2] studies the development of LBS from the perspective of communication and believes that the integration of LBS and social media exists in two forms: one is a special LBS social networking site and the other is a kind of LBS technology formed by other social networking sites. *Social Communication Mode*. In the integration process of LBS and network media, the user privacy protection, information authenticity, and market demand still need to be adjusted and avoided [3]. Literature [4] made a detailed analysis of the advantages and disadvantages of LBS interpersonal communication and compared it with the real interpersonal relationship. It was proposed that the LBS interpersonal communication model would lead to prominent alienation, affect normal interpersonal relationships in reality, and reduce real-life interpersonal relationships. Interpersonal skills, increased trust crisis, degraded interpersonal responsibility, and even LBS social interactions will become criminal tools for criminals. Reference [5] puts forward corresponding improvement suggestions to promote the healthy development of LBS interpersonal communication and interpersonal relationships. Another research perspective is to explore LBS from the perspective of business services. Literature [6] proposes that location-based business information services have quietly emerged in China, and how to connect businesses with the needs of surrounding consumers is a solid foundation for the development of LBS. Reference [7] provides insights and predictions on the future development trend of LBSNS by studying the information acquisition, sharing, privacy protection of social network location services, and user identification and location recognition. Literature [8] analyzes the feasibility of applying LBS to the group buying industry and discusses the existing problems and suggestions for improvement of the group buying website based on LBS. Literature [9] summarizes and analyzes the mobile e-commerce marketing model based on LBS based on relevant cases in the field of mobile e-commerce and predicts the development trend of mobile e-commerce based on LBS. Literature [10] proposed the prospect of mobile development of LBS business and the strategy of LBS application innovation through the SWOT analysis model and carried out a simple LBS system planning and design for the industrial application of LBS personal products with practical needs. Reference [11] builds an LBS group buying business adoption model and verifies the hypothesis that perceived trust, perceived usefulness and ease of use, and network externalities are important factors that affect the willingness to use LBS group buying. Literature [12] uses theoretical analysis tools and data analysis reports of mobile operators and consulting companies to analyze and study the development status, influencing factors, profit models, and development trends of the LBS industry, promotes the development of the LBS industry, and provides suggestion on characteristics of electronic services.

There are not many studies on user behavior in my country. Scholars have studied the development of LBS from the user's perspective through different theoretical perspectives and discussed it in depth. Reference [13] evaluates the importance of specific quality elements from the perspective of user perception and proposes priority improvement directions for operators. Literature [14] put forward four hypotheses about the attitude and behavior of LBS information users and obtained relevant conclusions by sending out questionnaires to college students to collect data and analyze them. Literature [15] introduces the theory of self-construction, proposes a model of self-construction for users to accept mobile location services, and verifies it; Literature [16] uses social capital theory to analyze the impact of LBS's interpersonal communication on individual network capital, information capital, credit capital, emotion, and influence of capital. Reference [17] introduces influencing factors such as individual conformity into the original model of TAM users, builds a new hypothesis model, verifies the hypothesis, and puts forward suggestions for the development of the mobile location service industry. Reference [18] combines information system success theory. Combined with the information system success theory, the influence of information quality and system quality on perceived usefulness and ease of use is proposed, and a new research model of influencing factors of mobile location service usage intention is constructed. Literature [19] researches and analyzes users' consumption patterns from the perspective of location data and completes an intelligent system that integrates event detection, event prediction, and estimation of the number of customers. Reference [20] studies the user check-in data of LBSNS, analyzes and predicts the user behavior from the aspects of space, time, and social interaction, and establishes a location prediction model by using the main factors that affect the user's mobile behavior obtained by the study.

## 3. Social Network Information Service Based on User Behavior Perception

The perceptual data coverage optimization process is shown in Figure 1.

Participants collect perception data according to their own will. If the willingness of the participants is low, it means that the enthusiasm of the participants to perform the perception task is not high. Obviously, the service quality of the participants is low at this time, so it is necessary to measure the willingness of the participants. We assume that the set of participants is *N*={*n*_1_, *n*_2_,…, *n*_*r*_}. Considering that MCS is often used in scenarios with strong real-time and high complexity, we assume that *S*={*s*_1_, *s*_2_,…, *s*_*j*_} is the set of perception tasks divided by the platform according to factors such as time and geographic location. In addition, if we assume that participant *n*_*i*_ performs perception task *s*_*j*_, then the start time of perception task *s*_*j*_ is *t*_*s*_^*j*^, the end time is *t*_*e*_^*j*^, and *t*_*e*_^*j*^ − *t*_*s*_^*j*^ is the perception period of task *s*_*j*_. If *n*_*i*_ starts to perform perception task *s*_*j*_ at a time of *t*_*i*_^*j*^, then obviously the value range of *t*_*i*_^*j*^ is [*t*_*s*_^*j*^, *t*_*e*_^*j*^], and the decision time *h*_*ij*_ of *n*_*i*_ to perception task *s*_*j*_ is *t*_*i*_^*j*^ − *t*_*s*_^*j*^. If the time *t*_*i*_^*j*^ at which *n*_*i*_ starts to perform the perception task is closer to the start time *t*_*s*_^*j*^ of the perception task, then *n*_*i*_ is more motivated to perform the perception task, thus having a higher degree of willingness. In addition, there may be a one sidedness in measuring participants' willingness by a single factor, so the remaining battery power of participants' mobile devices is also considered here. If the remaining power value *V*_*i*_^*r*^ of the mobile device of the participant *n*_*i*_ is larger, then *n*_*i*_ has more willingness to perform the perception task without affecting the use of the mobile device, and the higher is the willingness of *n*_*i*_ at this time. Therefore, the willingness of the participants to perform the perception task *s*_*j*_ can be measured according to the participant's decision time *h*_*ij*_ for the perception task *s*_*j*_ and the remaining power *V*_*i*_^*r*^ of the mobile device. When the participant starts to perform the perception task at the same time as the start time of the task, the decision time *h*_*ij*_ of *n*_*i*_ to *s*_*j*_ at this time is 0, which means that the participant performs the task immediately when the task starts. Therefore, the willingness *W*_*ij*_ of the participants can be judged to be 1. To sum up, the quantification method of participants' willingness *W*_*ij*_ is shown in formula (1):

(1) $$\begin{array}{c} W_{ij}=\left\{\begin{array}{cc} \min\left\{\left[\frac{V_{i}^{r}}{V_{i}^{a}}\cdot \frac{h_{ij}}{\left(\sum_{i=1}^{v}h_{ij}/v\right)}\right],1\right\} & h_{ij}\neq 0,\\ 1, & h_{ij}=0. \end{array}\right. \end{array}$$

Among them, *V*_*i*_^*a*^ represents the total power of the mobile device, *v* represents the total number of participants performing the perception task *s*_*j*_, and *h*_*ij*_/(∑_*i*=1_^*v*^*h*_*ij*_/*v*) represents whether the decision time of participant *n*_*i*_ for *s*_*j*_ is lower than that of other participants.

Considering the temporal and spatial characteristics of the participant's movement trajectory, the participant's regional preference is not only related to the number of times the participant performs the perceptual task at the same regional location but also to the duration of the participant's perceptual task at the regional location. We assume that the region location of perceptual task *l*_*j*_ is *s*_*j*_. In the historical perception task list of participant *n*_*i*_, if *n*_*i*_ performs perception tasks at regional location *l*_*j*_ more times and the duration of the task is longer, then participant *n*_*i*_ has a greater preference for regional location *l*_*j*_. Moreover, the next time the perception task of the regional location *l*_*j*_ is performed, the more the real-time validity of the perception data can be guaranteed, and the higher the service quality of the participant *n*_*i*_ at this time. If participant *n*_*i*_ is performing the perception task for the first time, then the historical perception task list of *n*_*i*_ is empty at this time, so the platform sets the regional preference of *n*_*i*_ to 0, indicating that *n*_*i*_ has no regional preference.

If history-aware task list of *n*_*i*_ is nonempty, then in the history-aware task, the more times *l*_*j*_ performs the perception task, and there is the longer the duration of staying at the region location *l*_*j*_ during the execution of the perception task. At this time, it means that the regional preference *R*_*i*_^*l*_*j*_^ of the participant is larger. The participant's regional preference *R*_*i*_^*l*_*j*_^ is measured in terms of the number of times the participant performed the perceptual task at *l*_*j*_ and the duration of the perceptual task performed. In addition, considering that the number of times *n*_*i*_ performed perceptual tasks in *l*_*j*_, the duration of performing perceptual tasks has different degrees of influence on participant *n*_*i*_'s regional preference *R*_*i*_^*l*_*j*_^, and the calculation method of *R*_*i*_^*l*_*j*_^ is as follows:

(2) $$\begin{array}{c} \left\{\begin{array}{c} f_{1i}^{l_{j}}=\frac{O_{i}^{l_{j}}}{O_{i}},\\ f_{2i}^{l_{j}}=\frac{\sum_{o_{i}^{l_{j}}}\left(g_{i}^{l_{j}}-y_{i}^{l_{j}}\right)}{\sum_{o_{i}^{l_{j}}}\left(e_{i}^{l_{j}}-s_{i}^{l_{j}}\right)},\\ R_{i}^{l_{j}}=\alpha_{1}^{l_{j}}f_{1i}^{l_{j}}+\alpha_{2}^{l_{j}}f_{2i}^{l_{j}}. \end{array}\right. \end{array}$$

Among them, *f*_1*i*_^*l*_*i*_^ and *f*_2*i*_^*l*_*j*_^ represent the number of times *n*_*i*_ performs the perception task and the duration of the perception task at *l*_*j*_, respectively, and *O*_*i*_^*l*_*i*_^ is the number of times that *n*_*i*_ performs the perception task at the regional location *l*_*j*_. *O*_*i*_ is the total number of times the participant performs the perceptual task, and *y*_*i*_^*l*_*i*_^ and *g*_*i*_^*l*_*j*_^ are the time when *n*_*i*_ starts and ends the perceptual task in the regional location *l*_*j*_, respectively. *s*_*i*_^*l*_*i*_^ and *e*_*i*_^*l*_*j*_^ are the start time and end time of the perception task at region location *l*_*j*_, respectively. In addition, the weight *α*_1_^*l*_*j*_^ represents the degree of influence of *f*_1*i*_^*l*_*j*_^ on *R*_*i*_^*l*_*j*_^, *α*_2_^*l*_*j*_^ represents the degree of influence of *f*_2*i*_^*l*_*i*_^ on *R*_*i*_^*l*_*j*_^, and *α*_1_^*l*_*j*_^+*α*_2_^*l*_*j*_^=1.

In order to objectively reflect the influence of *f*_1*i*_^*l*_*i*_^ and *f*_2*i*_^*l*_*i*_^ on *R*_*i*_^*l*_*j*_^, this section uses the entropy weight method to calculate *α*_*g*_^*l*_*j*_^, *g*=1,2. At the same time, considering the difference in data dimension and order of magnitude between *f*_1*i*_^*l*_*i*_^ and *f*_2*i*_^*l*_*i*_^, it may bring errors in the calculation of *α*_*g*_^*l*_*j*_^. Therefore, we first normalize *f*_1*i*_^*l*_*i*_^ and *f*_2*i*_^*l*_*i*_^, as shown in the following formula:

(3) $$\begin{array}{c} \tilde{f_{gi}^{l_{i}}}=\frac{f_{gi}^{l_{j}}-\mu_{g}^{l_{j}}}{\sigma_{g}^{l_{j}}},\;g=1,2,\;i=1,2,\ldots ,\phi . \end{array}$$

Among them, *ϕ* is the number of participants who have performed perception tasks at regional location *l*_*j*_ in historical perception activities, and *ϕ*⊆*N*. In addition, *μ*_*g*_^*l*_*j*_^ and *σ*_*g*_^*l*_*j*_^ represent the mean and standard deviation of *f*_*gi*_^*l*_*j*_^, *g*=1,2, respectively, as shown in the following formula:

(4) $$\begin{array}{c} \left\{\begin{array}{c} \mu_{g}^{l_{j}}=\frac{\sum_{i=1}^{\phi }f_{gi}^{l_{j}}}{\phi },\\ \sigma_{g}^{l_{j}}=\sqrt{\frac{\sum_{i=1}^{\phi }{\left(f_{gi}^{l_{j}}-\mu_{g}^{l_{g}}\right)}^{2}}{\phi -1}},\;g=1,2. \end{array}\right. \end{array}$$

Second, in order to obtain the information entropy of *f*_*gi*_^*l*_*j*_^, first, according to formula (3), the proportion *φ*_*si*_^*l*_*j*_^ of *f*_*gi*_^*l*_*i*_^ after normalization can be obtained, that is, $\varphi_{gi}^{l_{i}}={\tilde{f_{gi}^{l}}}^{\tilde{l}}/\sum_{i=1}^{\phi }\tilde{f_{gi}^{l}}$. Then, the information entropy *H*_*g*_^*l*_*j*_^ of *f*_*gi*_^*l*_*i*_^ is obtained according to *φ*_*gi*_^*l*_*j*_^, as shown in the following formula:

(5) $$\begin{array}{c} H_{g}^{l_{j}}=\frac{\left(\sum_{i=1}^{\phi }\varphi_{gi}^{l_{j}}\ln\;\varphi_{gi}^{t_{j}}\right)}{\left(-\ln\;\phi \right)}. \end{array}$$

Finally, the weight of *f*_*gi*_^*l*_*i*_^ is obtained according to the entropy weight *β*_*g*_^*l*_*j*_^, corresponding to the information entropy *H*_*g*_^*l*_*j*_^ of *f*_*gi*_^*l*_*i*_^, as shown in the following formula:

(6) $$\begin{array}{c} \left\{\begin{array}{c} \beta_{g}^{l_{j}}=\frac{\left(1-H_{g}^{l_{j}}\right)}{\left(\sum_{g=1}^{2}1-H_{g}^{l_{j}}\right)},\\ \alpha_{g}^{l_{j}}=\frac{\beta_{g}^{l_{j}}}{\left(\sum_{g=1}^{2}\beta_{g}^{l_{j}}\right)}. \end{array}\right. \end{array}$$

The higher the willingness *W*_*ij*_ of *n*_*i*_, the more actively *n*_*i*_ participates in the perception task, and the more effectively the real-time perception data can be guaranteed. At this time, the service quality *M*_*i*_ of *n*_*i*_ is larger, so the willingness degree *W*_*ij*_ of *n*_*i*_ is proportional to *M*_*i*_, that is, *dM*_*i*_/*dW*_*ij*_ > 0:

(7) $$\begin{array}{c} M_{i}=\;\log_{2}\left(\frac{W_{ij}}{\max\left(W_{ij}\right)}+1\right),\;\forall n_{i}\in N. \end{array}$$

If participant *n*_*i*_ is not performing the perception task for the first time, then the service quality *M*_*i*_ of *n*_*i*_ needs to be measured according to its willingness and regional preference, so the service quality of *n*_*i*_ is as follows:

(8) $$\begin{array}{c} M_{i}=\;\log_{2}\left(\frac{W_{ij}}{\max\left(W_{ij}\right)}\cdot \frac{R_{i}^{l_{j}}}{\max\left(R_{i}^{l_{i}}\right)}+1\right),\;\forall n_{i}\in N. \end{array}$$

We assume that in each perception task, participants need to submit data *Q*={1,2, ⋯, *q*} times. Participants only need to go to the corresponding target points to collect perception data. In addition, in actual situations, the amount of perceptual information provided by the target points is not the same, so it is assumed that *ω*_*P*_*j*__={*ω*_1_, *ω*_2_,…, *ω*_*p*_} is the weight of *P*_*j*_, and *ω*_1_+*ω*_2_+⋯+*ω*_*p*_=1. Obviously, when the participant *n*_*i*_ has not yet started to perform the perception task *s*_*j*_, the value of *C*_*s*_*j*__^*q*^(*n*_*i*_) is 0 at this time. When *n*_*i*_ starts to perform perceptual task *s*_*j*_, as the number of target points covered by *n*_*i*_'s perceptual data increases, the perceptual coverage also increases. Therefore, the perceptual data coverage of participant *n*_*i*_'s q-th submission is shown in the following formula:

(9) $$\begin{array}{c} C_{s_{j}}^{q}\left(n_{i}\right)=\frac{\sum \omega_{m_{i}}m_{i}}{P_{j}}. \end{array}$$

Among them, *m*_*i*_ is the number of target points contained in the data perceived by participant *n*_*i*_, and *ω*_*m*_*i*__⊆*ω*_*P*_*j*__.

We assume that the set *λ*, *λ*⊆*N* of participants *f* submits perceptual data about task *s*_*j*_ for the q-th time. If the perception data submitted by participants *n*_*i*_ and *n*_*j*_ contain the same target points, then the same target points are considered only once when calculating the perception data coverage. Therefore, the coverage of the participant set *λ* is shown in the following formula:

(10) $$\begin{array}{c} C_{s_{j}}^{q}\left(\lambda \right)=\frac{1}{P_{j}}\left(\sum \omega_{e_{j}}e_{j}+\sum \omega_{y_{j}}y_{j}\right),\;\forall \omega_{e_{j}},\omega_{y_{j}}\in \omega_{P},\;\forall e_{j},y_{j}\in P_{j}. \end{array}$$

Among them, *e*_*j*_ represents the same target point in the participant set *λ* and *y*_*j*_ represents different target points.

We assume *U*_*s*_*j*__(*χ*) to be the platform's satisfaction. If the difference between *C*_*s*_*j*__(*χ*) and *δ*_*s*_*j*__ is small, then the value of *U*_*s*_*j*__(*χ*) is large. In addition, since *C*_*s*_*j*__(*χ*) and *δ*_*s*_*j*__ are represented in the form of matrices, this section uses the Frobenius norm to quantify the difference between *C*_*s*_*j*__(*χ*) and *δ*_*s*_*j*__ to evaluate the satisfaction *U*_*s*_*j*__(*χ*), as shown in the following formula:

(11) $$\begin{array}{c} U_{s_{j}}\left(\chi \right)=1-\frac{{\left\|\delta_{s_{j}}-C_{s_{j}}\left(\chi \right)\right\|}_{F}}{{\left\|\delta_{s_{j}}\right\|}_{F}}. \end{array}$$

Among them, ‖·‖_*F*_ represents the Frobenius norm.

It can be seen from the above that the platform not only needs to optimize the coverage of perception data. It is assumed that the utility of participant *n*_*i*_ is *ζ*_*s*_*j*__(*n*_*i*_). If the utility value *ζ*_*s*_*j*__(*n*_*i*_) of *n*_*i*_ is high, then the participant *n*_*i*_ not only guarantees the real-time validity of the perception data but also the coverage rate of the perception data when performing the perception task.

(12) $$\begin{array}{c} \zeta_{s_{j}}\left(n_{i}\right)=M_{i}\cdot \left[U_{s_{j}}\left(\chi +n_{i}\right)-U_{s_{j}}\left(\chi \right)\right]. \end{array}$$

Among them, *U*_*s*_*j*__(*χ*+*n*_*i*_) − *U*_*s*_*j*__(*χ*) represents the satisfaction of the participant *n*_*i*_ with the platform. If the satisfaction is high, then the perceptual data coverage of *n*_*i*_ is high.

We assume that the platform selects the perception data of the participant set S={*s*_1_, *s*_2_, ..., *s*_*j*_} for the perception task set *χ*^*∗*^. In order to maximize the utility of the participant set *χ*^*∗*^, this section first defines the perceptual data coverage optimization problem, as shown in the following formula:

(13) $$\begin{array}{c} \text{Maximize:}\zeta \left(\chi^{*}\right)={\left[\zeta_{s_{1}}\left(\chi^{*}\right),\zeta_{s_{2}}\left(\chi^{*}\right),\cdots ,\zeta_{s_{j}}\left(\chi^{*}\right)\right]}^{T},\\ \text{subject to:}\chi^{*}\subseteq N;\sum_{i\in \chi^{\prime }}f_{i}\leq J. \end{array}$$

When the utility of *ζ*_*s*,_(*χ*^*∗*^) increases, it needs to receive the perception data of more participants, so that formula (13) is converted into the following formula:

(14) $$\begin{array}{c} \text{Maximize:}\zeta \left(\chi^{*}\right)=\sum_{j=1}^{j}\frac{P_{j}}{\sum_{j=1}^{j}P_{j}}\zeta_{s_{j}}\left(\chi^{*}\right),\\ \text{subject to:}\chi^{*}\subseteq N;\sum_{i\in \chi^{\prime }}f_{i}\leq J. \end{array}$$

Among them, *P*_*j*_/∑_*j*=1_^*j*^*P*_*j*_ is the proportion of perception task *s*_*j*_. It will obviously affect the platform to select the number of participants' perception data, thus affecting the coverage of perception data. Therefore, according to the participant's utility and reward, the platform selects the participant's perception data with the highest reception efficiency in each iteration, and the efficiency *ϑ*(*n*_*i*_, *χ*^*∗*^) of participant *n*_*i*_ is shown in the following formula:

(15) $$\begin{array}{c} \vartheta \left(n_{i},\chi^{*}\right)=\frac{\left[\sum_{j=1}^{j}P_{j}/\sum_{j=1}^{j}P_{j}\zeta \left(\chi^{*}+n_{i}\right)-\sum_{j=1}^{j}P_{j}/\sum_{j=1}^{j}P_{j}\zeta \left(\chi^{*}\right)\right]}{f_{i}}. \end{array}$$

It can be seen from the above formula that if the reward of the participant *n*_*i*_ is higher, it will obviously affect the growth of the efficiency *ϑ*(*n*_*i*_, *χ*^*∗*^).

The proposed DCSQ strategy is validated by MATLAB, and the DCSQ strategy is compared with the IMRA strategy and the CrowdTasker strategy under different number of participants and different budgets. At the same time, the coverage rate, total perception time, and participants' total reward parameters under the three strategies are analyzed.

Figure 2 analyzes the effect of changes in perceived data coverage when the number of participants changes.

In Figure 3, it can be seen that with the increase in the number of participants, the total reward of participants changes according to the law of rapid growth at first and then almost stable. Compared with the CrowdTasker strategy, the DCSQ strategy also considers the real-time validity of the participants' perception data, so the total reward of the participants in the DCSQ strategy is the smallest.

Figure 4 compares the changes in the total perception time of the task for different numbers of participants.

The total reward of participants and the total perception time under different platform budgets are shown in Figures 5–7. Among them, Figure 5 reflects the changes in the perceived data coverage of the three strategies under different platform budgets. As the platform budget increases, the perception data coverage increases to a certain level and then remains stable.

In Figure 6, the total reward of participants increases first and then stabilizes as the platform budget increases. The reason is that as the platform budget increases, the platform chooses to receive more participant perception data. In Figure 7, as the platform budget increases, the total perception time first decreases and then slowly stabilizes.

## 4. Continuous Use Intention of Mobile Social Network Information Service Based on User Behavior Perception

Information quality, service quality, and system quality all have an impact on satisfaction. Therefore, in this study, the relationship between its two-dimensional variables and satisfaction is constructed. Because the information quality, system quality, and service quality are used as specific objective influencing variables to describe the user's postuse expectation, the expectation confirmation variable is deleted. The constructed user continuation intention model is shown in Figure 8(a).

From the perspective of user behavior perception, based on the ECM-ISC model, this study combines hedonic theory and herd theory to take perceived pleasure, imitating others, and not fully believing in the information they have as model variables. Moreover, this study introduces habit as a moderating variable between continuous use intention and behavior and constructs a continuous use model of mobile Internet-personalized service based on user behavior perception (Figure 8(b)). The model consists of two parts: the willingness model for continuous use of mobile Internet-personalized services and the model for continuous use behavior. In addition, it takes continuous use intention and continuous use behavior as dependent variables to study the effects of perceived pleasure and herding behavior on continuous use intention and the mechanism of user habits on continuous use intention and continuous use behavior.

On the basis of the above research, the continuous use intention of mobile social network information service based on user behavior perception is studied, and the effectiveness of the model in this study is calculated. The results are shown in Table 1. and Figure 9.

From the above systematic evaluation, it can be seen that the continuous use willingness system of mobile social network information service based on user behavior perception proposed in this study can basically meet the actual needs.

## 5. Conclusion

Mobile Internet-personalized service refers to providing users with mobile, ubiquitous personalized business services and information services according to the personalized and differentiated characteristics of users' information needs during the interaction process between users using mobile devices and servers, so as to meet the needs of users need. The utility of the mobile Internet-personalized service depends on the user's psychological cognition, acceptance, and use, and the user may continue to use the application only on the premise that the mobile Internet-personalized service is good. This study analyzes the continued use of mobile social network information services based on user behavior perception. Through algorithm research and systematic evaluation, it can be seen that the continuous use willingness system of mobile social network information service based on user behavior perception can basically meet the actual needs.

## Figures and Tables

**Figure 1:** Optimization process of data coverage.

**Figure 2:** Perceptual data coverage.

**Figure 3:** Total rewards for participants.

**Figure 4:** Total perception time.

**Figure 5:** Coverage.

**Figure 6:** Total rewards for participants.

**Figure 7:** Total perception time.

**Figure 8:** Continuous use intention of mobile social network information services based on user behavior perception (a) Continuous use intention model of user. (b) Personalized service continuous use intention model.

**Figure 9:** Statistical diagram of model evaluation.

**Table 1:** System model evaluation.

Number	Model evaluation
1	83.89
2	88.97
3	81.56
4	91.87
5	88.05
6	90.49
7	79.65
8	89.25
9	89.41
10	79.26
11	86.58
12	88.53
13	80.95
14	80.19
15	85.16
16	90.98
17	88.76
18	85.17
19	92.97
20	89.00
21	79.86
22	79.52
23	82.89
24	84.45
25	85.69
26	88.90
27	83.78
28	89.37
29	91.38
30	88.72
31	80.58
32	90.23
33	83.52
34	84.21
35	90.51
36	85.24
37	88.39
38	90.15
39	91.80
40	90.84
41	89.40
42	87.36
43	80.68
44	80.55
45	87.30
46	91.91
47	87.29
48	91.07

## Data Availability

The labeled dataset used to support the findings of this study is available from the corresponding author upon request.

## References

[1] Chen X., Zou D., Xie H., Wang F. L. (2021). Past, present, and future of smart learning: a topic-based bibliometric analysis. *International Journal of Educational Technology in Higher Education*.

[2] Chen Y., Yang M. (2020). Intelligent design based neural network model for measuring analysis of the college teachers’ teaching ability. *International Journal of Emerging Technologies in Learning (iJET)*.

[3] Yang Z., Huang Y., Jiang Y., Sun Y., Zhang Y. J., Luo P. (2018). Clinical assistant diagnosis for electronic medical record based on convolutional neural network. *Scientific Reports*.

[4] Kumar K., Haider M. T. U. (2021). Blended computation of machine learning with the recurrent neural network for intra-day stock market movement prediction using a multi-level classifier. *International Journal of Computers and Applications*.

[5] Liu X., Zhang Y., Bao F., Shao K., Sun Z., Zhang C. (2020). Kernel-blending connection approximated by a neural network for image classification. *Computational Visual Media*.

[6] Dalal S., Khalaf O. I. (2021). Prediction of occupation stress by implementing convolutional neural network techniques. *Journal of Cases on Information Technology*.

[7] Halverson L. R., Graham C. R. (2019). Learner engagement in blended learning environments: a conceptual framework. *Online Learning*.

[8] Liu J., Zhu K., Lu W., Luo X., Zhao X. (2021). A lightweight 3D convolutional neural network for deepfake detection. *International Journal of Intelligent Systems*.

[9] Cheung S. K. S., Wang F. L., Kwok L. F. (2021). The continuous pursuit of smart learning. *Australasian Journal of Educational Technology*.

[10] Liu X., Xia Y., Yu H., Dong J., Jian M., Pham T. D. (2020). Region based parallel hierarchy convolutional neural network for automatic facial nerve paralysis evaluation. *IEEE Transactions on Neural Systems and Rehabilitation Engineering*.

[11] Yuan X., Elhoseny M. (2019). Intelligent data aggregation inspired paradigm and approaches in IoT applications. *Journal of Intelligent and Fuzzy Systems*.

[12] Ojala R., Vepsäläinen J., Hanhirova J., Hirvisalo V., Tammi K. (2019). Novel convolutional neural network-based roadside unit for accurate pedestrian localisation. *IEEE Transactions on Intelligent Transportation Systems*.

[13] Yin Z., Wu P., Foody G. M. (2020). Spatiotemporal fusion of land surface temperature based on a convolutional neural network. *IEEE Transactions on Geoscience and Remote Sensing*.

[14] Betere J. I., Kinjo H., Nakazono K., Oshiro N. (2020). Investigation of training performance of convolutional neural networks evolved by genetic algorithms using an activity function. *Artificial Life and Robotics*.

[15] Zhang J., Pan S., Hong H., Kong L. (2019). Blending ensemble of fine-tuned convolutional neural networks applied to mammary image classification. *Journal of Medical Imaging and Health Informatics*.

[16] Ferraz P. A. P., Oliveira B. A. G., Ferreira F. M. F., Martins C. A. P. d. S. (2020). Three‐stage RGBD architecture for vehicle and pedestrian detection using convolutional neural networks and stereo vision. *IET Intelligent Transport Systems*.

[17] DeLatte D. M., Crites S. T., Guttenberg N., Yairi T. (2019). Automated crater detection algorithms from a machine learning perspective in the convolutional neural network era. *Advances in Space Research*.

[18] Yao K., Unni R., Zheng Y. (2019). Intelligent nanophotonics: merging photonics and artificial intelligence at the nanoscale. *Nanophotonics*.

[19] Yang Z., Yang J., Rice K., Hung J.-L., Du X. (2020). Using convolutional neural network to recognize learning images for early warning of at-risk students. *IEEE Transactions on Learning Technologies*.

[20] Sreenu G., Durai M. A. S. (2019). Intelligent video surveillance: a review through deep learning techniques for crowd analysis. *Journal of Big Data*.

